# Integration and Optimization of British and American Literature Information Resources in the Distributed Cloud Computing Environment

**DOI:** 10.1155/2022/4318962

**Published:** 2022-06-07

**Authors:** Mei Chen

**Affiliations:** Nanchong Vocational and Technical College, Nanchong 637000, China

## Abstract

One of the most effective approaches to improve resource usage efficiency and degree of resource collecting is to integrate resources. Many studies on the integration of information resources are also available. The search engines are the most well-known. At the same time, this article intends to optimize the integration of British and American literature information resources by employing distributed cloud computing, based on the needs of British and American literature. This research develops a model for the dispersed nature of cloud computing. It optimizes the method by fitting the mathematical model of transmission cost and latency. This article analyzes the weaknesses of the current British and American literature information resource integration and optimizes them for the integration of British and American literature resources. The Random algorithm has the longest delay, according to the results of this paper's experiments (maximum user weighted distance). The algorithms NPA-PDP and BWF have longer delays than the algorithm Opt. The percentage decline varies between 0.17 percent and 1.11 percent for different algorithms. It demonstrates that the algorithm presented in this work can be used to integrate and maximize information resources from English and American literature.

## 1. Introduction

In the past ten years, cloud computing has experienced rapid development and has been widely used. Many commercial cloud computing service providers (cloud service providers, CSPs) began to provide a variety of public cloud computing services. More enterprises and organizations have also built their own private cloud infrastructure or built hybrid cloud facilities. Achieving efficient utilization and management of cloud computing resource pool resources can not only reduce service costs, but also improve service quality and competitiveness. The current problem is how to allocate resources to meet the service quality requirements of diversified businesses, reduce costs, and increase profits. Therefore, resource allocation is one of the most basic and core issues in cloud computing service deployment.

At the same time, the research on British and American literature is becoming more and more enthusiastic, and the demand for British and American literature resources is increasing. Whether it is a literary worker or the general public, the thirst for literary knowledge is getting higher and higher. However, the resources of British and American literature are widely distributed in archives, websites, and libraries around the world, which makes it difficult and costly to obtain. In addition, the language of British and American literature includes Old English, confused language, and other mixed languages, which are not easy to read. Therefore, combined with the characteristics of distributed cloud computing, it is necessary to integrate and optimize the global British and American literature resources.

The main innovations of this paper are as follows: it optimizes the delay and cost of migrating distributed big data of British and American literature to the cloud. Firstly, the selection target of data center during data migration is analyzed. It proposes an approximate algorithm for fair data placement and optimal data placement. It simultaneously extends the traditional k-supplier problem, the capacity-unlimited facility location problem, and the k-middle point problem. Aiming at the two goals of minimizing data placement for transmission cost and minimizing data placement for total cost, a nearest data center priority heuristic algorithm is proposed. The proposed algorithm can effectively reduce latency, save costs, and solve the problem that some data centers are unavailable due to regulatory restrictions or user preferences during data migration.

## 2. Related Work

In order to maximize the profits of CSPs and optimize the user experience, in recent years, it has become a trend to use multiple cloud networks to provide services in a unified manner. In the multi-cloud structure, cloud broker service has been recommended as a basic cloud service and has attracted extensive attention from industry and academia. Tsai and Lo proposed an efficient distributed mobile cloud computing service authentication scheme. His scheme reduces the authentication processing time required for communication and computation between cloud service providers and traditional trusted third-party services. Formal security proofs and performance analysis show that the scheme is both secure and efficient [1]. Hirai et al. modeled the task scheduling server as a single-server queue, where the server consists of many workers. When a task enters the server, the task is split into subtasks. Each subtask is served by its own worker and an alternate different worker [2]. Xiong et al. believed that, with the rapid development of mobile services, mobile cloud computing (MCC) has received great attention from researchers in academia and industry. He will design an enhanced and provably secure authentication scheme for distributed MCC services [3]. Kakade et al. eliminated the need for an uninterruptible power supply (UPS) in the data center by connecting direct current voltage from a backup power source directly to the motherboards of multiple servers in the data center. The alternating current power received from the electric utility service is converted to a lower voltage by on-site transformers and then supplied to one or more power distribution units on-site [4]. Liao et al. proposed an active data prefetching scheme on the storage server of the distributed file system for cloud computing. Experiments demonstrate that their proposed active prefetching technique can benefit distributed file systems in cloud environments to achieve better I/O performance [5]. Deng et al. proposed a distributed intrusion detection based on hybrid gene expression programming and cloud computing (DID-HGEP Cloud) for the massive and high-dimensional intrusion data behavior in cyber-physical power systems. Through comparative experiments, it is shown that the algorithm they proposed has obvious advantages in false attack rate, DAR, average time consumption, etc. Furthermore, the proposed algorithm has excellent parallel performance [6]. Alhazmi et al. believed that cloud computing provides on-demand IT services through large distributed data centers on high-speed networks. Virtualization is a key cloud computing technology. It allows service providers to offer computing services in a cloud environment without platform compatibility differences. He formulated the virtual network configuration in a geographically distributed cloud computing data center supporting SDN as a mixed integer linear programming (MILP) problem. The formulation of the proposed Optimal Virtual Network Provisioning (OVNP) model is studied by simulation. The experimental results verify the effectiveness of his proposed method [7]. However, through the summary of related research, it can be found that although the current research on distributed cloud computing is very in-depth, there is no research on resource integration for British and American literature. This is detrimental to the development of the resource integration of English and American literature in China.

## 3. Distributed Cloud Computing

Cloud computing has become the preferred platform for big data analysis [8, 9]. Especially when data is generated from multiple geographically distributed locations, local users need to use local data frequently, and sometimes all local data need further joint analysis. Therefore, it is more appropriate to use a cloud platform. For example, for a multinational sales company with many subsidiaries around the world, subsidiaries in each country need to analyze data generated by local users in a timely manner for business purposes. At the same time, all data should be aggregated and analyzed to report to headquarters or support cross-border transactions. For example, US demographic data is stored by state. Huge remote sensing data are stored in data centers across regions. Although these data are managed regionally, they may also require collaborative analysis for a common goal [10, 11]. Generally speaking, large-scale cloud computing is networked in a distributed manner. It has multiple geographically distributed data centers (Amazon has at least 11 DC1s across 4 continents; Google has at least 13 DC2s across 4 continents). Each DC configures computing and storage resources on a pay-as-you-go basis. This kind of infrastructure can provide nearby services and is especially suitable for data processing distributed across regions.

In order to process big data in cloud computing, the prerequisite is to migrate and store the data on a suitable data center (DC) [12]. Moving hardware directly is an optional way to move large-scale data. The Amazon Import/Export service, for example, recommends using removable storage devices to transport data, and sometimes it is even possible to move entire machines. But this is only suitable for infrequent, or one-time, bulk data movement. This method has a large delay and cannot meet the growing demand for real-time analysis of data. It also contradicts the idea of automated management and requires more labor participation. Transferring data over the Internet is very expensive and impractical due to the large delays. For example, it takes roughly 13 days to transmit 1 TB of data through a 10 MB internetwork. It is generally recommended to transfer real-time data over a high-speed dedicated connection (such as AWS Direct Connect1), which can speed up the transfer. But even relying on high-speed dedicated connections, transferring data across continents is difficult. For example, AWS Direct Connect does not provide cross-continental service, and international private lines are too expensive. This limits the movement of all large-scale data across the globe to the same DC [13, 14]. Also, using a DC to store data results in more frequent local data analysis delays. Especially in some regions, data security laws require that some data must be stored locally (e.g., some countries in the European Union). All in all, it is necessary for users to follow some rules to choose a suitable storage location for their data. As Amazon suggests, being closer to the user can reduce latency in data usage, meet specific legal and regulatory requirements, or reduce costs, etc.

Figure 1 simulates the distribution of DCs and users (for simplicity, users are used to represent subsidiaries or data owners).

There are a total of 10 DCs and 9 users in Figure 1, spanning 4 continents. Different users can use different DC services or prefer different DCs. For example, users 4, 5 in Europe can only be scheduled to DC5, 6 in Europe. Users in Asia only prefer DCs in Asia Pacific.

Cross-DC data analysis is now possible with various MapReduce-based frameworks, such as G-Hadoop and G-MR [15, 16]. A lower-cost cross-data center big data processing method is also proposed in this research. Using numerous DCs instead of just one can meet the needs of comprehensive data analysis while also ensuring faster local data analysis and cheaper expenses.

Considering the underlying incomplete graph,

(1) $$\begin{array}{c} G=\left(U,V,E\right). \end{array}$$

Among them, the side length

(2) $$\begin{array}{c} e_{ij}\in E,\;\left(i\in U,j\in V\right). \end{array}$$

It satisfies trigonometric inequalities, as well as positive integers *k*(*k* ≤ |*U*|, *k* ≤ |*V*|). This chapter aims to find a DC subset *D* (|*D*| ≤ *k*) from the available DC set V to store the data of all users in U according to different goals. For any *i* ∈ *U* and *j* ∈ *V*, if user i's data can be moved to DC *j* (at least not restricted by regulations or excluded by users), there is an edge between them. This problem assumes that all *i* are adjacent to at least one *j*; otherwise the problem has no solution. Also it assumes that

(3) $$\begin{array}{c} \left|E\right|=m. \end{array}$$

Among them,

(4) $$\begin{array}{c} m\leq \left|U\right|*\left|V\right|. \end{array}$$

Each user is assigned a weight *w*_*i*_, which represents the activation level of current or foreseeable future data generation, or the importance of local users. *w*_*i*_ increases with the amount of data or the importance of the user. The activation level rather than the data volume is used because it can tolerate the dynamic changes in the data while providing a modest approximation to the data volume. The activation level can be based on the amount of data uploaded per day. For example, for a typical company uploading 200 GB per day [17], 10 GB can be used as the threshold for determining the activation level. If a subsidiary generates less than 10 GB of data per day, a weight of 1 can be assigned. For subsidiaries between 20 and 30 GB, a weight of 3 is assigned. By analogy, for user *i* with activation level *w*_*i*_, a fee *w*_*i*_*e*_*ij*_ will be charged to move data to DC *j*.

Each DC has a different price for compute and storage resources. For more economical storage and processing of data, lower prices are of course preferred. Given DC *j*, assume that the price of one VM instance processing data per hour is *a*_*j*_. On average, such instances are able to analyze *b*_*j*_ GB of data per hour. Then, the price for processing 10 GB of data is

(5) $$\begin{array}{c} p_{j}^{\prime }=\frac{10*a_{j}}{b_{j}}. \end{array}$$

If the storage cost for 10 GB of data is *p*_*j*_′′, then the total cost on the DC side for a user with activation level 1 is

(6) $$\begin{array}{c} p_{j}=p_{j}^{\prime }+p_{j}^{\prime \prime }. \end{array}$$

For user *i* with activation level *p*_*j*_′, if it wants to store and process data at DC *j*, it needs to pay *w*_*i*_*p*_*j*_.

Because of the high scalability of cloud computing, this chapter assumes that the DC has no computing and storage capacity constraints. For data integrity, a user's data is only stored in one DC. The target data center selection problem can be summarized as follows: it selects at most *k* target DCs and assigns each user to a target DC such that it satisfies the following objectives.

Fair data placement (FDP): the maximum distance between the user and the assigned DC is minimized so that each local user can access data with minimal delay:

(7) $$\begin{array}{c} \min\;D\subseteq V,\left|D\right|\leq k^{\max};i\in U,j\in D\left(e_{ij}\right). \end{array}$$

Preferred data placement (PDP): the maximum weighted distance between the user and the assigned DC is minimized, allowing local users with more data to access data with minimal delay:

(8) $$\begin{array}{c} \min\;D\subseteq V,\left|D\right|\leq k^{\max};i\in U,j\in D\left(w_{i}e_{ij}\right). \end{array}$$

If needed, it also uses

(9) $$\begin{array}{c} w\left(i,j\right)=w_{i}e_{ij}, \end{array}$$

to represent the weighted distance.

Transmission cost minimization data placement (TCMDP): transmission cost is defined as the minimization of the sum of the weighted distances between all users and the DC to which they are assigned:

(10) $$\begin{array}{c} \min\;D\subseteq V,\left|D\right|\leq k\left(\sum_{i\in U}j\in D\left(w_{i}e_{ij}\right)\right). \end{array}$$

Total cost minimization (cost minimization data placement, CMDP): the total cost is defined as the minimization of the sum of the costs for all users:

(11) $$\begin{array}{c} \min\;D\subseteq V,\left|D\right|\leq k\left(\sum_{i\in U}j\in D\left(c_{ij}\right)\right). \end{array}$$

It needs to note that goal 1 is a special case of goal 2 when *w*_*i*_ = 1. Goal 3 is a special case of Goal 4 when *p*_*j*_ = 0, and subsequent discussions will focus on goals 2 and 4. The corresponding results can be directly applied to objectives 1 and 3, respectively.

Suppose *x*_*ij*_ is a Boolean variable that indicates whether user *i* is assigned to DCj. It is 1 if *i* is assigned to *j*, and 0 otherwise. *y*_*j*_ is also a Boolean variable that indicates whether DCj is used. It is 1 if used, and 0 otherwise.

The PDP problem wants to minimize the largest weighted distance *z*, where

(12) $$\begin{array}{c} w_{i}e_{ij}x_{ij}\leq z\;\forall i\in U,j\in V. \end{array}$$

PDP can be formalized as the following 0–1 mixed integer program:

(13) $$\begin{array}{c} \begin{array}{c} \min z\\ \text{s.t} \end{array}, \end{array}$$

(14) $$\begin{array}{c} \sum_{j\in V}x_{ij}=1,\;\forall i\in U, \end{array}$$

(15) $$\begin{array}{c} y_{j}\geq x_{ij}\;\forall i\in U,j\in V, \end{array}$$

(16) $$\begin{array}{c} x_{ij}\in \left\{0,1\right\},y_{j}\in \left\{0,1\right\}, \end{array}$$

(17) $$\begin{array}{c} x_{ij}=0\text{ for some }i\in U,j\in V. \end{array}$$

Constraint (13) guarantees that every user must be assigned to at least 1 DC. Constraint (14) guarantees that this DC must be used. And the number of selected DCs cannot exceed *k* (Constraint (15)). Moreover, not all DCs can be used by every user (Constraint (16)); that is, the underlying bipartite graph is incomplete.

CMDP can be formalized as the following 0–1 integer linear program:

(18) $$\begin{array}{c} \begin{array}{c} \min\sum_{i\in U,j\in V}\left(w_{i}e_{ij}+w_{i}p_{j}\right)x_{ij}\\ s.t\;\left(13\right),\left(14\right),\left(15\right),\left(16\right),\left(17\right) \end{array}. \end{array}$$

In the objective function, both *e*_*ij*_ and *p*_*j*_ are in normalized form. The first half ∑_*i*∈*U*,*j*∈*V*_*w*_*i*_*e*_*ij*_*x*_*ij*_ is the transmission cost. The second half, ∑_*i*∈*U*,*j*∈*V*_*w*_*i*_*e*_*ij*_*x*_*ij*_, is the cost of storing and processing data in the data center.

PDP is an extension to the k-vendor problem, while CMDP is a common extension to the UFL and k-middle point problem. Because of the k-vendor problem, both UFL and k-middle point problems are NP-insoluble [18, 19]. So both PDP and CMDP are NP-insoluble. This section presents an approximation algorithm for PDP and a heuristic algorithm for CMDP. For the convenience of reading, the special summary abbreviation table is shown in Table 1.

## 4. Strategies and Methods for Integrating Information Resources of British and American Literature

### 4.1. Engine Search Aspects

The search engine is mainly composed of four parts, namely, the information collector (robot or spider or crawler), the analysis indexer (indexer), the searcher (searcher) and the query interface. The composition and structure of the current mainstream search engines generally include miners for data mining and user information mining [20]. Its connection mechanism is shown in Figure 2:

The availability of engine search is poor, and it is difficult to cope with the challenge of information islanding. The countermeasures include improving the ranking of mainstream engine search and improving the daily management system of engine search by improving the intelligent search engine. One of the major reasons why users cannot find the information they need is that they are not familiar with literature classifications; that is, users may not understand the classification information of English and American literature websites. Or the literary works recommended by the website are too professional, so that users cannot find the information they need when searching in plain language.

A better solution is to filter the correspondence between the vernacular words and the official words according to semantic analysis and probability statistics by collecting the search keywords of users on British and American literature websites. And according to the corresponding relationship, a lexicon of common people is generated. After receiving the vernacular words input by the user, the intelligent search engine system will query the Baiqiao style thesaurus, obtain official words matching the vernacular words input by the user, and search the website according to the obtained official words. Intelligent guidance, keyword association, and other technologies used in business engines such as Baidu are widely used to intelligently correct and sort retrieval results, so as to facilitate user retrieval. At the same time, box calculation can also be used to optimize the user's search results. The difference between this approach and the traditional approach is that, in the traditional search, users need to filter the search results. This kind of search system displays application services on the search result page by formulating association rules and engine search application containers.

When users use the search system to retrieve the information they need, they often do not search the system through the engine on the homepage of the English and American literature website but directly retrieve the required information in the mainstream search engine. Therefore, the search for British and American literature can improve the ranking of website information resources by purchasing services on mainstream engines such as Baidu. It can learn from the relatively mature engine search optimization guidelines in the United States and the United Kingdom and strive to enhance the visibility of information resources.

In the engine search of English and American literature websites, the latest search is empty, the information resource structure is single, and the update is not timely, which will cause the poor search function of the engine. Therefore, this article recommends that an experienced and first-class technical information management professional team be responsible for the maintenance of the search system, and to update and maintain the system in time. At the same time, English and American literature websites can consider using information integration and real-time monitoring procedures for user experience to achieve automatic integration and manual integration, daily integration and emergency integration, individual integration, and coordinated integration. In this way, a complete management chain such as real-time information monitoring, crisis early warning, and emergency response can be realized, and the search ranking of information resources on Chinese English and American literature websites can be improved.

In the face of the impact of emerging information technologies such as big data and the threat of information islanding, the website management department should put the needs of citizens first. This is also the core of the new public service theory; that is, the engine search design of the website should be more humanized and intelligent. The website content should show more hotspots that are closely related to civic life. The management department should take citizen satisfaction as the basis for evaluating website performance. Open data should be more concerned with fulfilling citizens' needs for specific data. On this basis, website management can consider strengthening the top-level design to improve the information resource management system. Website management should continue to improve the intensive construction of infrastructure, avoid duplication of construction, and improve the efficiency of equipment use.

### 4.2. Content Integration of British and American Literature

Internet search and information disclosure are the core and private content of Chinese British and American literature websites. It examines website content integration from the perspective of web search. It conducts an online survey on the online search services of English and American literature websites across the country. The current network search services are summarized as follows: (1) based on the account of the English and American literature website at the same level, the Internet search service of Bukou is integrated. The main feature of this model is that the service interface is unified and easy to integrate. However, this form of integration only guides users to the websites of various ministries, districts, and counties through address links for online search service requirements and does not actually integrate service resources on a unified platform. (2) Relying on brick-and-mortar bookstores, the online center at the same level is integrated. The advantage of this mode is to provide users with a unified login entry, and to realize the combination of the front-end service and the back-end service system; that is, the English and American literature website already has a service system. However, there are problems such as inconsistency in the handling process and service content between the newly built service integration platform and the already built service integration platform.

From the angle of information disclosure of English and American literature websites, the integration of website content is investigated. By analyzing the search, download, and reading usage of British and American literature websites, it finds that the biggest shortcoming is that although the number of British and American literature websites has been increasing actively, the number of applications for disclosure has not decreased accordingly but has continued to increase. In the software evaluation, the websites of districts and counties within the range of 600 were also tested. It found that about 90% of the websites were blocked and the updates were not timely enough. More than 80% of the websites have the phenomenon that the page cannot be opened or the function cannot be used. 90% of websites have fake links, dark links, and unusable links. The operation, maintenance, and management of grassroots websites need to be improved.

### 4.3. Open Data Integration of British and American Literature

The evaluation report on the construction of English and American literature websites of the State Information Center believes that, in the construction of open data, the situation of information islanding is serious. In a research evaluation of the practice of open data on British and American literature websites across the country, it was found that, as of May 2019, 86.25% of the data were updated annually or not at all. Only 13.75% of the data are updated monthly or daily.

From the problems of open data platforms, it can be seen that the number of data applications provided by open data platforms in various places is poor. Although some platforms have opened data application channels, the existing “applications” on the platform are not downloadable and useable data applications, but only the results of functional tests. Although some platforms provide downloadable and useable data applications, most of them do not use the data of this site or only use basic data such as geographic location in a shallow level. Or even if the data of this site is used, it does not explain which data is used. Some platforms offer “data apps” that do not live up to their name. In fact, it is the business processing system of local literature, and it is the source of open data, not the practical application after data opening, which greatly dampens the enthusiasm and creativity of users.

First of all, many British and American literature websites lack the awareness of change and do not realize the impact of big data and other information technologies on Chinese British and American literature websites. The main problem is that information technology such as big data is only understood as a common technical means. It did not realize that big data would improve the integration efficiency of information resources of English and American literature websites and promote the reform of literature administration. Many developers are not clear about the trend of e-government reform such as open data and even have resistance. Developers' awareness of technological innovation needs to be enhanced. Secondly, it is difficult for the laws and regulations of China's informatization standards to keep up with the pace of technological change. The laws and regulations of electronic technology informatization and big data construction are relatively lagging behind. The information integration of Chinese English and American literature websites requires the personnel in charge of British and American literature websites to strengthen the top-level design, enhance the efficiency of Chinese big data to promote the information integration of British and American literature websites, and improve the pertinence of problems. Finally, the talent construction of Chinese English and American literature websites cannot meet the impact of big data and other information technologies. The phenomenon of insufficient innovative talents and professional and technical talents, low level of internationalization of talents, and serious loss always exists. The key reason lies in the disconnection between China's e-government personnel training system and selection system. This requires China's public service department to reform its management system, select the right talent in an unorthodox way, and break down the identity barrier. Only in this way can it form an open, inclusive, and orderly pattern of talent selection.

## 5. British and American Literature Information Resource Integration System

Aiming at the problems existing in English and American literature websites and search platforms, this paper focuses on three aspects: engine search optimization, content integration optimization, and public information integration optimization. Combined with the low cost and high efficiency of distributed cloud computing, combined with the problems of wide distribution of English and American literature websites and many kinds of languages, it optimizes the experiment and cost of the website.

### 5.1. Optimization of Engine Search

To evaluate the impact of DC size on the BWF algorithm, it is assumed that users 1∼9 can be served by different numbers of candidate DCs. It adds one DC at a time to DCs 1∼10 in order from 11 to 14. The performance of each algorithm is shown in Figure 3.

As shown in Figure 4, the time delay (maximum user weighted distance) of the Random algorithm is the largest. The delays of the algorithms NPA-PDP and BWF are larger than those of the algorithm Opt. First, the algorithms NPA-PDP and BWF both choose DC2, 6, 9. When the number of DCs increases from 10 to 13, the delays of the algorithms NPA-PDP and BWF and the assignment relationship from users to DCs are the same. This is because none of the 3 DCs added subsequently are better than the preceding DCs, so none of the 3 DCs are chosen. When DC14 (Beijing) is added, the delays of algorithms NPA-PDP and BWF both increase. The reason is that user 8 (Xian) has the largest user weight, so the algorithm selects it as the user representative for the Asia-Pacific region. Because user 8 is closest to DC14 (Oakland), the algorithm abandons DC9 and chooses DC14 instead. Users originally assigned to DC9 are reassigned to DC14. This causes the delay to rise as the weighted distance between Beijing and Oakland.

The Opt. algorithm has the smallest delay. Although the number of DCs has increased, the delay has remained the same. Although the delay solved by the BWF algorithm is slightly larger than that solved by the Opt. algorithm, the average is about 5%. Experiments show that the Opt. algorithm can only optimize the main objective function value but cannot optimize the delay of other clusters. For example, the algorithms NPA-PDP and BWF both choose DC2, 6, and 9. Algorithm Opt. chooses 2, 5, 7. Among the three algorithms, the users served by DC2 are the same, namely, users 1, 2, and 3. NPA-PDP and BWF assign users 4, 5 to DC6. And Opt. assigns them to DC5. Users 6, 7, 8, and 9 are assigned to DC9 by algorithms NPA-PDP and BWF, and assigned to DC7 by algorithm Opt. The delays for each user are compared in Table 2. Obviously, the total delay of the Opt. algorithm is larger than that of the other two algorithms. This is because the Opt. algorithm cannot consider all clusters.

The experiment also increased the number of users from 9 to 19. It joins two users at a time in numerical order. The delay results are shown in Figure 5.

When users 18, 19 join, the delay changes because their minimum weighted distance is greater than the current delay. This also reveals that even if the number of users increases, it is not necessary to use more DC. Only when more distant users join is it possible to cause greater delays and thus require more DCs. Although the Opt. algorithm finds the optimal solution, the experiment again observes that the total delay of the Opt. algorithm is larger than that of the BWF algorithm. Although limited by the randomness of user location selection, a purely increasing delay curve cannot be drawn, but the simulation results still reveal a trend: the delay will not decrease as users join.

It is worth noting that when users 12 and 13 join in, the delay of NPA-PDP algorithm increases sharply. This is because the NPA-PDP algorithm simply deletes a DC without considering the user's grouping attributes. This also reflects the instability of NPA-PDP algorithm.

In terms of running time, Random algorithm and NPA-PDP algorithm are faster than the other two algorithms. All in all, the Opt. algorithm requires more time than the BWF algorithm. With the addition of DCs and users, the time consumption of the Opt. algorithm increases rapidly. The time consumed by the BWF algorithm is much slower, so it is more suitable for large-scale applications.

### 5.2. Content Integration and Optimization

In order to make full use of the various dimensions of PM resources, this section introduces the “similarity” boxing mechanism.  Figure 6 reveals the effectiveness of this mechanism. Simulation experiments are carried out for three scenarios, and the three sets of experiments include 450, 900, and 1500 VMs, respectively. In each set of experiments, the residual resources of each dimension of PM used were compared in the order of network bandwidth (N), CPU (C), memory (M), and hard disk storage (D). It can be seen from Figure 6 that the algorithm achieves a balanced use of resources in each dimension.

In order to save resource costs without compromising quality of service requirements, this section formalizes the problem as a stochastic multi-objective nonlinear programming. It targets a common situation (that is, VMs can be independent or related, and PMs can be heterogeneous and networked in a tree topology), while optimizing server and network bandwidth, which account for most of the data center cost. VM partitioning, statistical multiplexing, and “similarity” methods are used to implement a new offline algorithm and a new online algorithm. The effectiveness of the algorithm is verified through extensive simulation experiments. Experiments show that the algorithm proposed in this section is more effective. Not only do they drastically reduce PM and network-related resource costs, but they also guarantee a suitable quality of service.

### 5.3. Integration and Optimization of Public Information

The number of PM in each DC follows a U(3050) distribution. And the type of PM is uniformly chosen from four options. PM's configuration is based on the IBM SystemxM5 and Systemx3300M4 server types. The resource configuration requirements of the VMs in this chapter are based on the setup of four types of VMs from Amazon EC2's m3-series (for consistency with PM, GB is used to replace GiB). The M3-series is the most representative and is designed for general use. The number of logical cores per PM is equal to or at most twice the number of physical cores, according to VMWare8. The number of logical cores in a PM cannot exceed the number of vCPUs in a VM. Assume that vCPUs and physical cores have a one-to-one connection; the details are provided in Table 3.

Table 4 reflects resource pricing as well. Experiments strive to use Amazon as much as possible to expose data in order to maintain prices consistent. Because of the complex interaction between PM setup and VM resource requirements, only the medium type resource pricing is shown here. The prices of the remaining categories are expected to have the same multiplier relationship; for example, the price of xLargeVM with 4 vCPUs is four times that of the medium type. The pricing for storage is from Amazon S3. It may be computed that transferring 1 GB of data costs $0.0243 using the Amazon Import/Export service pricing.

TLGGA convergence is seen in Figure 7 when there are four DCs (DC1DC4). The value of the objective function decreases rapidly and the curve is highly steep in the first 200 iterations (including crossover, mutation, and local optimization of all populations), according to simulation experiments. The curve begins to flatten down over the next 800 cycles. The goal function value declined extremely slowly after roughly 1,000 times, despite the fact that the method took longer. In less than two seconds, a good solution can be found.

There is a similar convergence pattern for different numbers of DCS. The cost values for 1,000 and 10,000 iterations are shown in Figure 8. It demonstrates that multiple repetitions do not result in a proportional reduction in the goal value. The decrease in percentage was merely 0.17 percent to 1.11 percent.

The use of Reducer deployment in Hadoop for big data processing across data centers is examined in this study. It first formalizes the challenge as a two-tier plan to keep expenses down and follow typical Hadoop localization principles. Layer 2 planning can take into account the co-selection of a DC and a server at the same time. The new architecture is then used to offer a novel cross-data center large data processing technique based on key distribution. The Reducer can be deployed to the DC with the greatest data to process and the lowest cost of other resources with this approach. Finally, the system is implemented using a two-layer grouping genetic algorithm (TLGGA). The approach employs a local optimization strategy and a customized starting population creation mechanism. TLGGA's efficiency is demonstrated through simulation results. It outperforms both the baseline Hadoop method and the most recent G-MR algorithm.

## 6. Conclusion

This paper focuses on the global British and American literature websites and studies the resource allocation algorithm in distributed cloud computing. Firstly, based on the sequence of cloud computing service deployment, it adopts the top-down engineering theory method to divide cloud computing deployment into three stages: cloud network selection, data center selection, and server selection. Then, based on the specific business, it systematically studies the resource allocation methods in cloud computing according to the different goals and resources required by the business in each stage. Resource allocation based on distributed cloud computing still has many problems to be solved. The next step will focus on the research of distributed cloud computing algorithm.

## Figures and Tables

**Figure 1:** Data centers and users distributed across geographies.

**Figure 2:** Search engine basic structure process.

**Figure 3:** Comparison of the maximum delay obtained by the algorithm when the number of DCs increases.

**Figure 4:** Comparison of algorithm running time when the number of DCs increases.

**Figure 5:** Comparison of the maximum delay obtained by the algorithm when the number of users increases.

**Figure 6:** Physical node cost.

**Figure 7:** Convergence of TLGGA with 4 DCS.

**Figure 8:** Cost comparison for different iterations of different numbers of DCS.

**Table 1:** Algorithm abbreviation correspondence table.

Name	Abbreviate
Fair data placement	FDP
Preferential data placement	PDP
Transmission cost minimization data placement	TCMDP
Cost minimization data placement	CMDP

**Table 2:** Opt. algorithms cannot optimize every cluster.

User	BWF	Opt.
User 4	6679	25189
User 5	5137	23172
User 6	17893	9496
User 7	18542	54108
User 8	38263	88790
User 9	141337	134541

**Table 3:** PM resource configuration and VM resource requirements.

PM	Cores	Memory	VM	vCPUs	Memory
Medium	4	32	Medium	2	3.75
Large	8	64	Large	4	7.50
Xlarge	24	192	Xlarge	8	15.00
2xlarge	32	256	2xlarge	vCPUs	30.00

**Table 4:** Serial numbers and resource prices of data centers in different regions.

Data center location	California	Frankfurt	Singapore	Sao Paulo	Oregon	Ireland	Sydney
Medium PM	0.408	0.400	0.498	0.480	0.480	0.380	0.472
Medium VM	0.077	0.075	0.098	0.095	0.095	0.073	0.093
Save	0.033	0.0324	0.030	0.0408	0.0408	0.030	0.033
Power	11.910	9.490	15.470	14.370	14.370	8.900	15.470

## Data Availability

The data used to support the findings of this study are available from the author upon request.
